RETRACTED

# Immunohistochemistry Study of OY-TES-1 Location in Fetal and Adult Human Tissues

**DOI:** 10.1155/2022/7052830

**Published:** 2022-04-13

**Authors:** Jun Fu, Yingying Ge, Qingmei Zhang, Yongda Lin, Chang Liu, Weixia Nong, Xin Luo, Shaowen Xiao, Xiaoxun Xie, Bin Luo

**Affiliations:** ^1^Department of Histology & Embryology, School of Pre-clinical Medicine, Guangxi Medical University, Nanning 530021, China; ^2^Guangxi Colleges and Universities Key Laboratory Research of Preclinical Medicine, Guangxi Medical University, Nanning 530021, China; ^3^Department of Neurosurgery, First Affiliated Hospital, Guangxi Medical University, Nanning 530021, China

## Abstract

OY-TES-1 is reportedly involved in carcinogenesis and spermatogenesis. However, the tissue distribution of OY-TES-1 in the normal human body remains elusive. This study detected OY-TES-1 expression in human fetal and adult normal tissues by immunohistochemistry. We identified a general principle of OY-TES-1 expression. The expression of OY-TES-1 was found in neurons, smooth muscle cells, and cardiac muscle cells from both fetuses and adults. The connective tissue showed no specific staining throughout the fetal and adult samples. With OY-TES-1-positive staining of the epithelium irregular, OY-TES-1 was strongly expressed in the epithelium of the skin and bladder, as well as hepatocytes, pancreatic islets, and acinous cells during the fetal stage but was not detected in the postnatal period. In contrast to the epithelium of blood vessels, the fetal and adult central hepatic vein and glomeruli showed negative expression of the OY-TES-1 protein. Sex-dimorphism was observed in the distribution of OY-TES-1 in male and female germ cells. Collectively, our results indicate that OY-TES-1 is a member of the cancer-testis antigen and autoantigen, with tissue-specific and period-specific expression patterns, revealing potential contributions of OY-TES-1 to the diagnosis and therapeutic treatment for neoplasms and infertility.

## 1. Introduction

Cancer-testis antigens (CTAs) are a class of genes preferentially expressed in cancerous tissues and the testis [1]. In several species, including mice, pigs, guinea pigs [2], and stallions [3], OY-TES-1 has been detected in the acrosome of spermatozoa. A 32-kDa mature-type sperm protein (sp32) will be produced when the N-terminal half of OY-TES-1 is removed posttranslationally during spermatogenesis and/or sperm maturation [2, 4]. It has been reported that OY-TES-1 plays an important role in spermatogenesis and fertilization-related events [2, 5–8]. Whether these results apply to humans and whether there are species differences in OY-TES-1 function remains mysterious.

RETRACTED

Numerous studies have depicted abnormal expression of OY-TES-1 in many tumors such as epithelial ovarian cancer [9], colorectal cancer [10], and glioma [11] where its expression is associated with poor patient outcomes, high tumor grades, and malignant characteristics such as tumor cell invasion and metastasis. The production of OY-TES-1 was confirmed to induce an immune response by cytotoxic T cells *in vitro* [12, 13] or antibodies in cancer patients [9, 14–16]. Downregulation of OY-TES-1 was also noted to attenuate cell migration ability *in vitro* [17, 18].

Investigating the association between OY-TES-1 and human tissue differentiation and development is significant for exploring the mechanism underlying the role of OY-TES-1 in tumorgenesis. Therefore, in this paper, we aimed to detect the expression of OY-TES-1 in human fetal and adult normal tissues and compare its expression in tumors to provide further information on its functions.

## 2. Materials and Methods

### 2.1. Human Specimens

Tissue arrays of human fetuses (FeOrg-N090) at 19 weeks to 7 months and healthy organs (FDA808k-1) from adults aged 20 to 46 years, together with diagnosis reports, were obtained from Shanghai Outdo Biotech Company (Shanghai, China) and Xian Alenabio Company (Xian, China), respectively. The human fetal and adult tissues, normal adult testes, and ejaculated sperm used in our research were all collected with informed consent and following institutional ethics review board requirements. The organs detected were from the nervous, circulatory, immune, endocrine, digestive, respiratory, and urogenital systems (Table 1).

The present study was approved by the Medical Ethics Committee of Guangxi Medical University (approval number: GCMC201803120) and obtained patients' written informed consent.

### 2.2. Antibody Dilution

To optimize the working conditions of the antibody for immunohistochemistry analysis, rabbit preimmune and immune serum of OY-TES-1 protein were purified and adjusted to a concentration of 0.10 mg/ml. The immunohistochemical staining for tissue samples was performed at the same time. We determined the protein expression by combining the intensity score and the area core. The intensity level was defined as follows: 0, no staining; 1, weak staining; 2, moderate staining; and 3, strong staining. The area score was defined based on the percentage of positive cells as follows: 0, 0–5%; 1, 5%–25%; 2, 26%–50%; 3, 51%–75%; and 5, >75%. According to the sum of the intensity score and the area score, each section was assigned to negative expression (overall score = ‘-'), 0–1 point; weak expression (overall score = ‘+'), 2–3 points; moderate expression (overall score = ‘++'), 4–5 points; and strong expression (overall score = ‘+++'), 6–7 points. Positive immunoreactivity was evaluated by two experienced independent pathologists who were blinded to each other's assessments. If there is a contradiction between the evaluations of the two pathologists, estimation by a third pathologist was required. The optimal working dilution was determined by comparing the staining results with those in the Human Protein Atlas database (HPA039081 and HPA039082). Strong cytoplasmic staining was observed in a subset of cells in the seminiferous ducts and the acrosome of ejaculated sperm (https://www.proteinatlas.org/ENSG00000111644-ACRBP).

RETRACTED

### 2.3. Immunohistochemistry

Immunohistochemistry (IHC) analysis was performed as previously described [15]. After deparaffinization and rehydration, the tissues were incubated in 3% H_2_O_2_ for 10 min to block endogenous peroxidase activity, rinsed in Tris-buffered saline containing Tween 20 (TBST), and incubated twice for 10 min each time in TBST supplemented with normal goat serum to block nonspecific binding. The OY-TES-1 antibody was incubated in a humidified chamber overnight at 4°C. The tissues were incubated with the Supervision^TM^ horseradish peroxidase-conjugated goat anti-rabbit IgG (Zhongshan Jinqiao Biotech, Beijing, China) secondary antibody for 15 min at room temperature. Immunodetection was performed with 3, 3′-diaminobenzidine (Maixin Biotech, Fujian, China), and the samples were counterstained with hematoxylin. As a negative control, purified IgG from rabbits prior to immunization (original IgG concentration of 0.10 mg/ml) was diluted to corresponding ratios (1 : 500, 1 : 1000, and 1 : 1500), respectively.

## 3. Results

### 3.1. Optimization of Dilution of OY-TES-1 Antibody

Three working dilutions (1 : 500, 1 : 1000, and 1 : 1500) of the OY-TES-1 polyclonal antibody (original IgG concentration of 0.10 mg/ml) were tested on human adult testis tissues and ejaculated sperm. While maintaining the other conditions, IHC was performed on normal adult testis tissue at different dilution ratios of the OY-TES-1 antibody. The Human Protein Atlas database showed the IHC results of OY-TES-1 in testicular tissue. When the working dilution of the OY-TES-1 antibody was 1 : 1500, the staining of the seminiferous tubules was very light. At a dilution of 1 : 500, strong and nonspecific staining was observed within the seminiferous tubules (data not shown). As shown in Figure 1, with the antibody diluted to 1 : 1000, spermatogenic cells showed a strongly positive reaction and Leydig cells had a less positive reaction. No reactivity was observed in Sertoli cells. For ejaculated sperm, the acrosome presented highly OY-TES-1 specifically staining (Figure 1(c)). These results are consistent with those in the Human Protein Atlas database. Therefore, a 1 : 1000 dilution is the optimal dilution of the OY-TES-1 antibody.

RETRACTED

### 3.2. Localization of OY-TES-1 in Human Fetal Organs

In the digestive tract, OY-TES-1 was detected in the esophagus (Figure 2(a)), stomach (Figure 2(b)), duodenum (Figure 2(c)), and colon (Figure 2(d)). The results showed that the immune staining was mainly located on the cytomembrane of epithelial cells and the cytoplasm of glandular cells, epithelial cells, and smooth muscle cells in these organs. Additionally, OY-TES-1 was absent in the connective tissue of these organs.

In the digestive gland, hepatocytes (Figure 3(a)) and epithelial cells of the interlobular artery, interlobular vein, and interlobular bile duct showed moderate expression of OY-TES-1 (Figure 3(a)). However, no signal was detected in the central vein (Figure 3(b)). In the pancreas (Figure 3(c)), stronger immunostaining appeared in the pancreatic islets rather than acini, with the weakest signal observed in the ductal epithelium.

In the respiratory system, the cytoplasm of epithelial cells in the respiratory tract and the cytomembrane of alveolar cells showed low to moderately positive signals (Figure 3(d)). Feeble staining of chondrocytes was detected in the respiratory tract, which was difficult to distinguish from non-specific staining (Figure 3(e)). In organs of the circulatory system, staining by the OY-TES-1 antibody was observed in the cardiomyocytes and endothelium of the blood vessels (Figure 3(f)).

In the urinary system, OY-TES-1 was highly expressed in both the epithelial cells and smooth muscle cells of the bladder (Figure 4(a)). OY-TES-1 was highly expressed in the cytoplasm of epithelial cells in both the proximal and distal tubules (Figure 4(b)). Remarkably, the expression of OY-TES-1 was negative in the glomerulus (Figure 4(c)) mainly composed of blood vessels.

In the fetal testis sample, the staining of cells in the seminiferous cord showed variable results. In the nucleus, some cells showed a high density of staining, whereas others exhibited moderate staining. Some of the cells in the seminiferous cord were OY-TES-1-negative (Figure 4(c)). Furthermore, OY-TES-1 was immunoassayed in the cytoplasm of Leydig cells, a type of endocrine cell (Figure 4(c)). In the fetal ovary, OY-TES-1 expression was positive in the cytoplasm and nucleus of primary oocytes in the primary follicle, whereas negative in the follicular cells (Figure 4(d)).

In the central nervous system, OY-TES-1 was highly expressed in the cytoplasm of neurons (Figure 5(a)). As shown in Figure 5(b), OY-TES-1 protein was found in the nerve fibers of the sciatic nerve rather than the perineurium consisting of connective tissue.

RETRACTED

Notably, OY-TES-1 protein was widely expressed in the glandular epithelium of the adrenal gland (Figures 5(c) and 5(d)), adenohypophysis (Figure 6(a)), and thymus (Figure 6(b)). Additionally, strong positive immunostaining was observed in the sweat gland, hair follicles, and stratified squamous epithelium of the skin (Figures 6(c) and 6(d)). As expected, the connective tissue in the skin was negative for OY-TES-1.

### 3.3. Localization of OY-TES-1 in Human Adult Organs

Furthermore, we intended to determine the localization of the OY-TES-1 protein in the adult tissue arrays (Figures 7–9). In the adult digestive tract, OY-TES-1 had a restricted expression in the mucosa epithelium of the stomach (Figure 7(a)), duodenum (Figure 7(b)), colon (Figure 7(c)), and esophagus (Figure 7(d)). In the digestive gland, no OY-TES-1 staining was observed in hepatocytes (Figure 7(e)), pancreatic islets, and acini (Figure 7(f)). OY-TES-1 expression was variable in the adult adrenal gland with low membrane expression in the zona glomerulus (Figure 8(b)) and no significant staining in the zona reticularis and zona fasciculate (Figure 8(a)). Similarly, adenohypophysis cells exhibited three expression patterns: cytoplasmic-positive, nuclear-positive, and completely negative staining patterns (Figure 8(c)). In contrast, OY-TES-1 was consistently expressed in alveolar epithelial cells (Figure 8(d)), neurons (Figure 8(e)), cardiac muscle cells (Figure 8(f)), and smooth muscle cells (Figures 7(a) and 7(d)).

In the adult kidney, OY-TES-1 was positive in the renal tubule and negative in the glomerulus (Figure 9(a)). IHC analysis of the adult testis confirmed that Leydig cells were OY-TES-1-positive. The OY-TES-1 expression in the testis was maintained in the fetal period (Figure 9(b)). Spermatogonia showed strong staining for OY-TES-1, mainly in the cytoplasm but diffused in the nuclei and cytoplasm of spermatocytes. For round and early spermatids, signals were restricted in a small or narrow part of the cytoplasm. As expected, OY-TES-1 protein expression was focused on the acrosome of the elongated or late spermatid. In the adult ovary, the primary oocyte in the primary follicle was positive for OY-TES-1 expression, and the surrounding follicle cells were negative (Figure 9(c)). The expression pattern was similar to that observed in the fetal ovary sample. In contrast, in the secondary follicle, the primary oocyte did not express OY-TES-1, whereas the surrounding follicle cells showed weak and focal expression (Figure 9(d)).

RETRACTED

## 4. Discussion

This is the first study to comprehensively characterize the OY-TES-1 protein in a large cohort of healthy fetal and adult tissues. Our data expand the understanding of the expression pattern of OY-TES-1 protein and support that OY-TES-1 is a tissue-specific autoantigen, which may help reveal the pathogenesis of neoplasms, hypoplasia, and infertility.

For IHC, the testicular tissue of healthy adults was used as a positive control. With the staining data of the adult testis from the Human Protein Atlas database as a reference, the optimal dilution of the OY-TES-1 antibody was determined to ensure the reliability of immunostaining results.

Both fetal and adult neurons showed the same strong staining pattern of OY-TES-1 expression. OY-TES-1 may be involved in the development of the embryonic nervous system and nervous activity in adulthood. A previous study showed that the level of OY-TES-1 expression in the cerebral cortex was altered after improving the learning and memory ability of mice [19]. OY-TES-1 is presumably involved in keeping the nervous system functioning properly. This hypothesis should be interpreted cautiously. In-depth research is very limited.

Our data confirmed that the OY-TES-1 antibody showed a consistently strong immune response in both the smooth and cardiac muscle cells of the fetus and adult. Both the muscle tissue and the connective tissue represent mesoderm-derived tissue. In contrast, the connective tissue of various organs was essentially negative for OY-TES-1 expression. These results show that the expression of OY-TES-1 is not strictly related to the origin of the germ layer but depends on the tissue type, indicating the diverse biological function of OY-TES-1.

Our results displayed three different staining patterns of OY-TES-1 in the seminiferous tubule of the fetal testis. In the adult seminiferous tubule, OY-TES-1 protein expression varied in the contiguous segments during spermatogenesis. This underscores the functional diversity and precise regulation of OY-TES-1 in spermatogenesis. Spermatids of OY-TES-1-null mice failed to form a large acrosomal granule, leading to the fragmented structure of the acrosome and, eventually, severely reduced fertility [20]. Anti-OY-TES-1 antibodies reduced porcine capacitation and spontaneous acrosome reactions, which were able to cause fertilization disorders [21]. It is meaningful to further investigate the physiological role of OY-TES-1 in human spermatogenesis. In the female reproductive system, the primary oocyte inside the secondary follicle expressed OY-TES-1 but not during development to the primary oocyte stage. The differences in the expression patterns of male and female germ cells suggest that the function of OY-TES-1 is sex-dimorphic. More research is needed to explore the function of OY-TES-1 in human fertility.

RETRACTED

These observations reveal that the development stages and cell types affect the location and intensity of OY-TES-1 expression. We found that OY-TES-1 was expressed in the mucosal epithelium of the digestive tract in both the fetal and adult periods. However, some exceptions were observed. In the fetus, OY-TES-1 was detected in the endothelium of blood vessels in most of the organs evaluated, except the central hepatic vein and capillaries of the glomeruli, the reasons of which are currently unclear to us. OY-TES-1 was expressed in fetal hepatocytes, pancreatic islets, and acinous cells but was lost in adulthood. It is generally accepted that the carcinogenic process is initiated before birth [22, 23]. Indeed, the expression of OY-TES-1 will be inhibited when a hepatocyte becomes cancerous [18]. The potential of OY-TES-1 as a tumor genotyping marker deserves further investigation.

Some poorly differentiated tumors, such as colorectal cancer, ovarian cancer, and glioma, were found to have higher OY-TES-1 expression than well-differentiated tumors or their adjacent tissues [10, 11, 15]. OY-TES-1 expression may be significantly higher in the tumors of ovarian cancer patients with shorter survival times and faster relapse than those with longer survival [24, 25]. Higher expression of OY-TES-1 appears to be related to high cell proliferative activity, as supported by several *in vitro* experiments [17, 18, 24]. In addition, the therapeutic and prophylactic effects of multiepitope vaccines containing OY-TES-1 were confirmed in ovarian cancer [26, 27]. Regular OY-TES-1 expression may maintain the high fidelity of normal cell mitosis. Conversely, ectopic OY-TES-1 expression may alter cell proliferation, causing disordered cell differentiation and, thus, triggering tumorigenesis. More research into this question is clearly needed.

The expression of OY-TES-1 in normal adult tissues has less restriction than other CTAs, suggesting that OY-TES-1 belongs to the testis-selective CTA subfamily [28]. OY-TES-1 was expressed both in distinct tissues of the fetus and adult, which indicates its potential as an autoantigen. It is believed that high OY-TES-1 expression or expression outside the normal location should be regarded as ectopic and a target of immunoreaction [29, 30].

Collectively, we showed that as a CTA, OY-TES-1 is an autoantigen with a tissue-specific and period-specific expression pattern, while OY-TES-1 may play a key role in normal tissue development, fertility, or cancer susceptibility. This study is beneficial to revealing the mechanism and potential prediction value of OY-TES-1 in dysplasia, infertility, and tumorigenesis.

RETRACTED

## Figures and Tables

**Figure 1:** Immunolocalization of OY-TES-1 in human adult testis tissue and ejaculated sperm. (a) Adult testis as the positive control. Red circle: seminiferous tubule; white arrow: spermatogonia; gray arrow: spermatocyte; black arrow: round and early spermatid; red arrow: elongated or late spermatid; black triangle: Sertoli cell. (b) Adult testis was incubated with purified IgG from rabbits prior to getting immunized as the negative control. Red circle: seminiferous tubule; white arrow: spermatogonia; gray arrow: spermatocyte; black arrow: round and early spermatid; red arrow: elongated or late spermatid; red triangle: Leydig cell; black triangle: Sertoli cell. (c) Ejaculated sperm was incubated with OY-TES-1 antibody. (d) Ejaculated sperm was incubated with purified IgG from rabbits prior to getting immunized as the negative control.

**Figure 2:** Immunolocalization of OY-TES-1 in human fetal tissue. (a) Esophagus. Red arrow: epithelium; white rectangle: smooth muscle. (b) Stomach. red arrow: epithelium; white rectangle: smooth muscle. (c) Duodenum. Red arrow: epithelium. (d) Colon. Red arrow: epithelium; white rectangle: smooth muscle.

**Figure 3:** Immunolocalization of OY-TES-1 in human fetal tissue. (a) Liver. Red triangle: hepatocyte; red arrow: interlobular artery; black arrow: interlobular vein; green arrow: interlobular bile duct. (b) Liver. Red triangle: hepatocyte; red arrow: central vein. (c) Pancreas. Red circle: pancreatic islet; black circle: acini. (d) Lung. Red arrow: epithelium of trachea; black arrow: epithelium of pulmonary alveoli. (e) Lung. White rectangle: chondrocyte. (f) Heart. White rectangle: cardiac muscle; red arrow: artery; black arrow: vein.

**Figure 4:** Immunolocalization of OY-TES-1 in human fetal tissue. (a) Bladder. Red arrow: epithelium. (b) Kidney. Red circle: glomerular; red arrow: proximal convoluted tubule; black arrow: distal convoluted tubule. (c) Testis. Red circle: seminiferous cord; red arrow: Leydig cell; black arrow: spermatogenic epithelium. (d) Ovary. Red circle: primary follicle; red arrow: primary oocyte; black arrow: follicular cell.

**Figure 5:** Immunolocalization of OY-TES-1 in human fetal tissue. (a) Spinal cord. Red arrow: neuron; white rectangle: nerve fiber. (b) Sciatic nerve. Red arrow: peripheral myelinated nerve fiber; white rectangle: perineurium. (c) Adrenal gland. White rectangle: zona reticularis. (d) Adrenal gland. White rectangle: zona glomerulosa; gray rectangle: zona fasciculata.

**Figure 6:** Immunolocalization of OY-TES-1 in human fetal tissue. (a) Adenohypophysis. Red arrow: glandular epithelium. (b) Thymus. Red circle: thymic corpuscle. (c) Epidermis. Red arrow: sweet gland; white rectangle: hair follicle. (d) Epidermis. White rectangle: epithelium.

RETRACTED

**Figure 7:** Immunolocalization of OY-TES-1 in human adult tissue. (a) Stomach. Red arrow: epithelium; white rectangle: smooth muscle. (b) Duodenum. Red arrow: epithelium; white rectangle: smooth muscle. (c) Colon. Red arrow: epithelium; white rectangle: smooth muscle. (d) Esophagus. Gray rectangle: epithelium; white rectangle: smooth muscle. (e) Liver. Red triangle: hepatocyte; red arrow: central vein. (f) Pancreas. Red circle: pancreatic islet; red arrow: acini.

**Figure 8:** Immunolocalization of OY-TES-1 in human adult tissue. (a) Adrenal gland. White rectangle: zona reticularis; gray rectangle: zona fasciculata. (b) Adrenal gland. Gray rectangle: zona glomerulosa. (c) Adenohypophysis. Red arrow: glandular epithelium. (d) Lung. Red arrow: epithelium of pulmonary alveoli. (e) Cerebella. Red arrow: neuron. (f) Heart. White rectangle: cardiac muscle; red arrow: artery.

**Figure 9:** Immunolocalization of OY-TES-1 in human adult tissue. (a) Kidney. Red circle: glomerular; red arrow: proximal convoluted tubule; Black arrow: distal convoluted tubule. (b) Testis. Red circle: seminiferous tubule; white arrow: spermatogonia; gray arrow: spermatocyte; black arrow: round and early spermatid; red arrow: elongated or late spermatid; red triangle: Leydig cell; black triangle: Sertoli cell. (c) Ovary. Red circle: primary follicle; red arrow: primary oocyte; black arrow: follicular cell. (d) Ovary. Red circle: secondary follicle; red arrow: primary oocyte; black arrow: follicular cell.

**Table 1:** Comparison of OY-TES-1 expression among tissues of human fetus and adult.

Tissues	Germ disk	Cells	Organs tested	Expression of OY-TES-1 in fetus	Expression of OY-TES-1 in adult
Nerve tissue	Ectoderm	Neuron	Brain and spine	+++	+
			Spinal	+	+
Epithelial tissue	Ectoderm	Simple squamous epithelium	Skin	+	+(HPA)
		Glandular epithelium	Skin	+++	N
	Entoderm	Alveolar cells	Respiratory tract	+	+
		Epithelium of mucosa	Digestive tract	+∼++	−/+
		Transitional epithelium	Bladder	+++	+(HPA)
		Thymic corpuscle epithelial cell	Thymus	+	N
		Hepatocyte	Liver	++	−
		Pancreatic islet and acini	Pancreas	++	−
	Mesoderm	Endothelium	Blood vessel	+ (Central vein, glomerular -)	+ (Central vein, glomerular -)
		Glandular epithelium	Adenohypophysis	+	−/+
			Adrenal gland	+∼+++	−/+
		Renal tubule	Kidney	++	++
		Leydig cell	Testis	+	+
		Spermatogenic cell	Testis	+∼+++	+∼+++
		Oocyte	Ovary	+	+ (Primary follicle) - (secondary follicle)
		Follicular cell	Ovary	−	− (Primary follicle) + (secondary follicle)
Muscle tissue	Mesoderm	Smooth muscle	Digestive tract	+++	+++
		Cardiac muscle	Heart	++	++
Connective tissue	Mesoderm	Fibroblast	Digestive tract	−	−
		Chondrocyte	Respiratory tract	−	−(HPA)

+: Weak expression; ++: moderate expression; +++: strong expression; −: negative; N: did not detected; HPA: data from the Human Protein Atlas.

RETRACTED

## Data Availability

The datasets used and/or analyzed during the current study are available from the corresponding author on reasonable request.
